# Emerging roles and underlying molecular mechanisms of DNAJB6 in cancer

This article has been retracted.

**DOI:** 10.18632/oncotarget.9803

**Published:** 2016-06-02

**Authors:** Erhong Meng, Lalita A. Shevde, Rajeev S. Samant

**Affiliations:** ^1^ Department of Pathology, University of Alabama at Birmingham, Birmingham, Alabama, USA; ^2^ Comprehensive Cancer Center, University of Alabama at Birmingham, Birmingham, Alabama, USA; ^3^ Beijing DOING Biomedical Technology Co. Ltd., Beijing,China

**Keywords:** DNAJB6, chaperone, cancer

## Abstract

DNAJB6 also known as mammalian relative of DnaJ (MRJ) encodes a highly conserved member of the DnaJ/Hsp40 family of co-chaperone proteins that function with Hsp70 chaperones. DNAJB6 is widely expressed in all tissues, with higher expression levels detected in the brain. DNAJB6 is involved in diverse cellular functions ranging from murine placental development, reducing the formation and toxicity of mis-folded protein aggregates, to self-renewal of neural stem cells. Involvement of DNAJB6 is implicated in multiple pathologies such as Huntington's disease, Parkinson's diseases, limb-girdle muscular dystrophy, cardiomyocyte hypertrophy and cancer. This review summarizes the important involvement of the spliced isoforms of DNAJB6 in various pathologies with a specific focus on the emerging roles of human DNAJB6 in cancer and the underlying molecular mechanisms.

## INTRODUCTION

Heat-shock proteins (Hsps) are key components of the cellular chaperone - co-chaperone network that prevent protein mis-folding and aggregation in the crowded intracellular milieu [1, 2]. Hsp40 and Hsp70 are two important groups of this family and they often function as interactors to execute distinct functions. Hsp40s (also known as DnaJ proteins) are defined by the presence of an approximate 70-amino-acid region known as the J-domain, which is responsible for interacting with the ATPase domain, and possibly the substrate-binding domain of its partner Hsp70 [3, 4]. On the basis of a survey of expressed sequence tag (EST) databases representing different mouse tissues and embryonic stages, more than 40 DnaJ/Hsp40-related genes are expressed in mammals [5, 6]. Besides their general function as chaperones, many Hsp40 proteins possess specific functions such as cell cycle regulation, transcriptional activation, signal transduction and tumor suppression [6-8].

DnaJ/Hsp40 homolog, subfamily B, member 6, also named mammalian relative of DnaJ (MRJ), is one of the members of DnaJB family and is ubiquitously expressed. It encodes a highly conserved member of the DnaJ/Hsp40 family of co-chaperone proteins that function with Hsp70 proteins to protect client proteins from irreversible aggregation during protein synthesis or during time of cellular stress [9]. In this article we describe the functional roles played by DNAJB6 in different pathophysiologies with a specific focus on its impact on cancer progression. We also bring forth the existence and known functional distinctions of its spliced isoforms.

## THE STRUCTURE, ISOFORMS AND DISTRIBUTION OF DNAJB6

Human DNAJB6 gene is mapped to the chromosome 7q36.3. There are two spliced isoforms of human DNAJB6; isoform a (2.5 kb transcript variant I, NM_058246) and isoform b (1.6 kb transcript variant II, NM_005494). Variant II differs in the 3' coding region and has a distinct 3' UTR, compared to transcript variant I [10]. The full length DNAJB6 isoform a [MRJ (L)] is comprised of 326 amino acids, whereas the shorter isoform b [MRJ (S)] has 242 amino acids. This short isoform lacks the carboxyl-terminal 95 amino acids compared to the large form but contains an additional 10 amino acids (KEQLLRLDNK). The significance of this amino acid stretch remains unexplored [11]. Apart from the differences at the carboxyl terminus, both isoforms share identical structure including a conserved N-terminal J domain, a G/F domain rich in glycine and phenylalanine residues and a C-terminal domain containing a serine-rich (“SSF-SST”) region. The N-terminal J domain is responsible for interacting with the constitutively expressed chaperone Hsp70. The SSF-SST region has been shown to be important for interactions with the transcription factor nuclear factor of activated T cells c3 (NFAT3c) and histone deacetylases (HDACs) and for DNAJB6 oligomerization [12]. The G/F domain of DNAJB6 has no specific function assigned but similar G/F domains of Hsp40 members have been suggested to participate in recognition of partially unfolded client proteins such as in bacterial DNAJ11-13 and yeast Sis1. The long isoform is predominantly localized to the nucleus, whereas the short isoform is predominantly cytoplasmic [13].(Figure 1)

**Figure 1:** Human DNAJB6 gene The genomic locus of human DNAJB6 gene is located on the long arm of q36.3 of chromosome 7 with 82,059 bases pairs in length. It is downstream of UBE3C, LOC777650, RPL36AP30 and upstream of LOC101927914 and LOC100506557. DNAJB6 has two transcript variants (I and II). Transcript variant I has 10 exons (2,494bp) while transcript variant II has 8 exons (1,568bp). Compared to transcript variant I, variant II differs in the 3' coding region and has a distinct 3' UTR. The full length DNAJB6 isoform a is comprised of 326 amino acids, whereas the shorter isoform b has 242 amino acids. The isoform b lacks the carboxyl-terminal 95 amino acids but contains an additional 10 amino acids (KEQLLRLDNK). Apart from the differences at the carboxyl terminus, both isoforms share identical structure including a conserved N-terminal J domain, a G/F domain rich in glycine and phenylalanine residues and a C-terminal domain containing a serine-rich (“SSF-SST”) region.

## DNAJB6's FUNCTIONS IN MULTIPLE DISEASES AND PHYSIOLOGICAL PROCESSES

Hsp70 and its Hsp40 (J-protein) co-chaperone partners provide broad protective effects. A major role of Hsp70 and Hsp40 is to prevent aggregation of misfolded proteins, but they also can protect cells from toxicity caused by amyloid-forming proteins without preventing formation of aggregates [14]. It is noted that co-chaperones are limiting nodes in a depleted chaperone network which maintains cellular proteostasis [15]. Various degenerative nervous system disorders such as Parkinson's disease, Alzheimer's disease, Huntington disease and various forms of dementia display pathological protein aggregation. Similarly pathological protein aggregation plays an important role in a variety of human myopathies [16]. DNAJB6 acts to prevent poly-Q dependent protein aggregation and cellular toxicity induced by the mutant huntingtin protein [17, 18]. This function of suppressors of poly-Q aggregation requires the C-terminal domain (amino acids 152-232). A differential role for the two isoforms of DNAJB6 has also been suggested by experiments demonstrating that DNAJB6a (the longer, nuclear- localized isoform) effectively suppresses nuclear poly-Q protein aggregation but is ineffective with cytoplasmic aggregation, while DNAJB6b (the shorter, cytoplasmic isoform) is a potent suppressor of cytoplasmic poly-Q aggregation [12]. DNAJB6 is also, present in the core of Lewy bodies and is highly up-regulated in astrocytes of patients with Parkinson's disease [19]. There, DNAJB6 has been shown to restore mitophagy by promoting the relocation of Parkin(C289G) and the autophagy marker LC3 to depolarized mitochondria [20]. However, it still remains to be explored if this upregulation is a cause or consequence of the disease.

Because DNAJB6 is ubiquitously expressed in various human tissues and implicated in other neurodegenerative diseases, it is interesting that patients with genetic mutations of DNAJB6 show a selective disease of muscle. The fact that DNAJB6 is a highly expressed DNAJB family member in skeletal muscle indicates its importance for its biologic importance to muscle tissue, yet at the same time it has contributed to the vulnerability of this tissue. This is due to the fact that DNAJB6-myopathy mutations are deleterious gain-of-function mutations [21]. A series of recent elegant studies convincingly showed that mutations within the G/F domain of DNAJB6 are a novel cause of dominantly-inherited myopathy [13, 22, 23]. For example, Limb-Girdle Muscular Dystrophy 1D (LGMD1D) is caused by mutations of DNAJB6. Mutations in amino acids Phe89, Phe91, Phe93 cause proximal LGM and mutations in Pro96, Phe100 of DNAJB6 cause distal-onset myopathy [21]. These mutations increase the half-life of DNAJB6 and reduce its protective anti-aggregation effect [13, 22, 24]. It is noteworthy that although the mutations alter the sequence of both nuclear and cytoplasmic DNAJB6, they affect muscle pathology exclusively through the cytoplasmic isoform [13]. Despite the documented prevalence of alternative splic­ing, the scientific literature contains few other such examples. Elucidation of the mechanisms by which certain isoforms of ubiquitously expressed mutant proteins can lead to organ-specific effects will be important for understanding genetic diseases and for developing therapeutic options [13]. Related to the focus of this review, the possible existence of these mutations in various malignancies and their functional relevance are still undetermined.

DNAJB6 has possible functional relevance to one more vital organ, the heart. Prolonged cardiac hypertrophy of pathologic etiology is associated with arrhythmia, sudden death, decompensation, and dilated cardiomyopathy. Extensive investigation to understand the mechanisms that underlie the hypertrophic response are centered on characterization of the molecular pathways that initiate or maintain the pathologic growth of individual cardiac myocytes. Calcium-calcineurin-NFAT-tumor necrosis factor α (TNFα) signaling pathway was shown to play an important role in regulating the cardiac hypertrophic response [25]. It has become increasingly clear that NFAT transcription factors are operative not only in T cells but control critical processes in many vertebrate developmental systems. Sustained activation of the Ca^2+^-calcineurin-NFAT signaling pathway has emerged as a powerful regulatory principle governing cardiac hypertrophy. In case of sustained Ca^2+^ increase and calcineurin activation, the calcineurin (a phosphatase) targets and dephosphorylates moderately conserved serine rich motifs at the N terminal homology region (NHR) of NFAT to unmask its nuclear localization signals. Subsequently, NFAT proteins shuttle into the nucleus where they accumulate on target promoter sites. TNF-α is a well-characterized downstream effector that directly responds through NFAT DNA binding sites within its minimal promoter [26]. Increased TNF-α expression is associated with a wide array of cardiac disease states including hypertrophy. MRJ reduces TNF- α expression by interacting with NFATc3 and histone deacetylase 4 (HDAC4), leading to the repression of calcineurin-induced cardiomyocyte hypertrophy [27] (Figure 3). Additionally interesting observations from Ding *et al* indicate that the long isoform of dnajb6b gene is important for late onset of cardiomyopathy in zebrafish and thus there may be more mechanistic details involving DNAJB6 in this disease to be unraveled [28].

**Figure 2:** DNAJB6 negatively regulates tumor growth and metastasis through Wnt signaling pathway Note: →indicates promotion and ┤indicates inhibition.

**Figure 3:** DNAJB6 represses cardiomyocyte hypertrophy through calcineurin-NFAT signaling pathway In case of sustained Ca^2+^ increase and calcineurin activation, NFAT proteins shuttle into the nucleus where they accumulate on target promoter sites. DNAJB6 reduces TNF- α expression through interacting with NFATc3 and HDAC4, leading to the repression of calcineurin-induced cardiomyocyte hypertrophy. Note: → indicates promotion; ┤indicates inhibition.

DNAJB6 also has been implicated in infectious viral diseases. It plays a role in the regulation of nuclear transport of pre-integration complex (PIC) of human immunodeficiency virus type-2 (HIV-2). The human and simian immunodeficiency viruses (HIV and SIV, respectively) have evolved the ability to productively infect non-dividing cells, a unique feature that distinguishes these lentiviruses from other retroviruses. This infection is mediated by active transport of the viral PIC into the nucleus without breakdown of the nuclear envelope during cell division. Components of the PIC that have been implicated in regulating nuclear import include the central DNA flap, as well as viral proteins IN, MA, and Vpr (HIV type 1 [HIV-1]) or Vpx (HIV-2 and SIV). Yeast two-hybrid screening performed by Cheng *et al*. identified that DNAJB6 interacts with Vpx. Overexpression of DNAJB6 specifically enhances the nuclear localization of Vpx whereas down-regulation of DNAJB6 by small interfering RNA (siRNA) reduces the nuclear import of these viral PICs [11].

Genomic DNA replication is an essential process for all herpesvirus including human cytomegalovirus. In the case of human cytomegalovirus (HCMV), DNAJB6 can also modulate the cellular distribution of the primase protein. HCMV UL70 protein, is believed to encode the primase activity of the viral DNA replication machinery and is highly conserved among herpesviruses. This protein needs to be localized in the nucleus which is the site of viral DNA synthesis. DNAJB6, was shown to specifically interact with UL70. The level of UL70 in the nuclei is increased in cells in which DNAJB6a is up-regulated or DNAJB6b is down-regulated, and is reduced in cells in which DNAJB6a is down-regulated or DNAJB6b is up-regulated. Furthermore, the level of viral DNA synthesis and progeny production was increased in cells in which DNAJB6a was up-regulated or DNAJB6b was down-regulated, and was reduced in cells in which DNAJB6a was down-regulated or DNAJB6b was up-regulated. Thus, DNAJB6a and b appear to influence the nuclear import and cytoplasmic accumulation of UL70. These suggest that the relative expression levels of DNAJB6 isoforms may play a key role in regulating the cellular localization of UL70, leading to modulation of HCMV DNA synthesis and lytic infection [29].

Recent studies by Taguwa *et al* revealed a key role of DNAJB6 in propagation of the mosquito-borne single positive-stranded RNA virus, the dengue virus (DENV), the cause of dengue fever. The chaperone-co-chaperone couple, Hsp70 and DNAJB6 together play a determinative role in the virion production by regulating protein assembly processes responsible to maintain viral proteostasis [30]. Thus the viruses seem to highjack the chaperoning activity of DNAJB6. This may possibly be applicable to more viruses and may emerge as a promising drug target.

In addition to the much reported relevance of DNAJB6 in diseases caused by protein aggregates, interesting roles of DNAJB6 isoforms have been implicated in embryonic development, intra flagellar transport and in influencing and determining the progression and outcome of multiple types of cancers [31-36].

## ROLE OF THE LONG ISOFORM OF DNAJB6 IN NEGATIVELY REGULATING TUMOR GROWTH AND METASTASES

Chaperones have long been suggested as important players in cancer biology [37-40]. Their roles range from regulation of cell cycle, transcription regulation, DNA repair, cell death mechanism, nucleosome integrity to mediation of response to environmental stress and ER stress [41-46]. Heat shock proteins 90 and 70 have gathered critical attention as therapeutic targets [47-51]. Multiple members of HSP40 family have also been suggested as important players in different aspects of tumor progression and metastasis [8, 52-61]. In this context, it is important to highlight the contributions of DNAJB6 in the pathology of this disease pathology.

Studies in breast cancer and melanoma cells led to the first functional elucidation of the role of DNAJB6a. This isoform has been shown to suppress tumorigenicity and metastasis of breast cancer cells. DNAJB6a levels are significantly reduced in aggressive breast cancer cells and in advanced grade infiltrating ductal carcinoma [34]. Over expression of DNAJB6a in aggressive breast cancer cell lines decreased their migration, invasion and reduced their motility. Its expression restricted orthotopic tumor xenograft growth in nude mice. Interesting mechanistic insight was obtained from the study of the secreted proteome of the DNAJB6a-expressing cells. These cells exhibited reduced levels of tumor progression and metastasis-promoting secreted proteins and increased levels of secreted metastasis suppressor [34]. Notably, these changes were registered in the transcript levels of these proteins. This implied a role of DNAJB6a in regulating signaling mechanism and transcription machinery that could impede tumor progression, a role that appeared overtly different from the implied chaperone functions.

Cell morphology studies revealed that DNAJB6a plays an important role in maintaining an epithelial-like characteristic in cancer cells. Expression of this isoform in invasive, mesenchymal-like cells causes changes in cell morphology concomitant with down-regulation of mesenchymal markers Vim (vimentin), CDH2 (N-cadherin), Twist1, and Slug (SNAI2) and up-regulation of epithelial marker keratin 18. DNAJB6a up-regulates dickkopf 1 homologue (DKK1), a secreted inhibitor of Wnt signaling [62, 63]. Thus inhibition of Wnt/β-catenin signaling is one of the molecular mechanisms by which DNAJB6a reverses epithelial mesenchymal transition (EMT) (Figure 2).

The intracellular signaling pathway activated by Wnts was originally identified as the β-catenin-dependent pathway (also referred as canonical Wnt pathway). This pathway is highly conserved among various species and is implicated in development, morphogenesis, stem cell maintenance, differentiation as well as wound healing. β-catenin is a cadherin-binding protein involved in regulation of cell to cell adhesion and is required to maintain epithelial morphology in association with its partner E-cadherin. Usually free β-catenin is ubiquitinated and rapidly degraded by proteosomal degradation. Axin acts as a scaffold protein to degrade β-catenin by forming a complex with glycogen synthase kinase 3β (GSK3β), β-catenin, adenomatous polyposis coli (APC) gene product, and casein kinase 1α (CK1 α). At low levels of β-catenin, the transcription factor TCF/LEF (T-cell factor /lymphocyte enhancer factor) binds to Groucho, which recruits HDACs to mediate transcriptional repression. However, once free from the membrane, β-catenin can translocate to the nucleus and function as an important mediator of Wnt signaling. In the presence of Wnt signaling, Wnts, such as Wnt1, Wnt3a, Wnt8, bind to cell-surface co-receptors consisting of Frizzled and LRP5/6. The cytoplasmic β-catenin is stabilized and enters the nucleus. In the nucleus, β-catenin associates with the basal transcriptional machinery, such as TATA box binding protein (TBP), and with transcriptional co-activators such as CREB-binding protein (CBP)/p300 and Brg1. By binding to TCF/LEF, β-catenin displaces Groucho to stimulate the transcription of target genes, including c-Myc, cyclinD1, Axin2, osteopontin (OPN), muscle segment homebox 1 (MSX1) [64-67]

The molecular mechanism of DNAJB6a's reversal of EMT is through activation of GSK3β. DNAJB6 chaperones a multiprotein complex DNAJB6a-HSPA8(HSP70)-PP2A. PP2A is a phosphatase that maintains GSK3β in a de-phosphorylated (active) state. Active GSK3β will prompt degradation of β-catenin. Thus β-catenin dependent transcription is down-regulated. MSX1 is a downstream target of β-catenin. Thus DNAJB6(L) compromises the expression of MSX1. Interestingly MSX1 is a transcription repressor of DKK1, a secreted inhibitor of Wnt signaling. Thus, lowered MSX1 levels up-regulate DKK1 production, resulting in a feed-forward repression loop that keeps a check on Wnt/β-catenin signaling [68, 69]. Evaluation of DNAJB6 levels from patient derived specimens helped define the disease relevance of these observations. DNAJB6 levels decrease significantly in invasive and metastatic breast cancer and melanoma [34, 68]. Thus it is tempting to speculate that in these patients the active state of GSK3β is compromised due to the lack of proper chaperoning of PP2A. This impairs degradation of free β-catenin, in turn allowing unrestricted Wnt/β-catenin driven transcription that can contribute to proliferation, invasion and EMT.

At this point it is necessary to highlight that DKK1 is among the best-characterized inhibitors of the canonical Wnt pathway [70]. However, DKK1 itself is a target gene of Wnt/ β-catenin signaling, thereby establishing a negative-feedback loop [71]. Thus, if Wnt signaling is on, DKK1 levels may increase to restore a check on Wnt signaling. However, MSX1 repression offers a Wnt/β-catenin driven repressive check on DKK1. It appears to be paradoxical to have the same signaling pathway upregulate and downregulate its repressor; in essence regulating a feed-back repression or a feed-forward activation loop. However, this emphasizes the intricate necessity for context dependent regulation of Wnt signaling and suggests a pivotal role of DNAJB6 as a checkpoint on Wnt/ β-catenin signaling (Figure 2).

Canonical Wnt signaling regulates cellular proliferation and differentiation. It is involved in many developmental processes as well as the development of tumors, such as colorectal cancer [66, 72]. Wnt signaling also regulates EMT [73, 74]. Though it is considered as a member of this pathway, GSK3β is a multifunctional kinase that regulates a critical signaling node of Wnt, Hedgehog and SNAIL signaling [65, 75]. Thus the activation of GSK3β mediated by DNAJB6a by chaperoning the DNAJB6a-HSPA8(HSP70)-PP2A tri-molecular complex has important implications in defining the details of signaling towards clinically targeting this node. As mentioned above, a typical DNAJ protein is characterized by a J domain, a glycine-Phenylalanine (G/F) domain and a C-terminal domain. Depending on the presence of these domains, this family is divided into Type I, Type II and Type III (also known as DNAJ A, B and C) types [76]. The J domain consists of highly conserved Histidine-Proline-Aspartic acid (HPD) tri-peptide and, is the most conserved domain of this family and has been implicated in providing the substrate specificity to the individual members [77]. The J domain of DNAJB6 is critical for its ability to restrict attributes of malignancy. Deletion of the J domain renders DNAJB6 incapable of dephosphorylating GSK3β consequently disabling it from targeting β-catenin for destruction [68].

Recent observations indicate a similar role of DNAJB6 in Esophageal Cancer (ESCC). Immunohistochemically Yu *et al* showed that nuclear localization of DNAJB6 is associated with survival of patients with esophageal cancer. Thus patients whose tumors showed high nuclear levels of DNAJB6 had a lower risk of death than patients with low levels of DNAJB6. Also, there was a negative association between the nuclear level of DNAJB6 and the presence of lymph node metastases [36]. Mechanistically it was shown that DNAJB6a reduced signaling through AKT. In many cancers, continuous activation of AKT signaling is a consequence of aberrant phosphorylation and thus activation of AKT1 at T308 and S473. These phosphorylation events are strictly controlled by multiple kinases and phosphatases. It was observed that the chaperoning of PP2A by DNAJB6a and Hsp70 plays a determinative role in AKT regulation. DNAJB6a complexes with HSP70/PP2A/AKT1 in the nucleus and promotes dephosphorylation of AKT1 by PP2A. From treatment perspective it must be noted that increasing DNAJB6a expression down-regulates AKT signaling but also decreases sensitivity to AKT inhibition. This suggests that ESCC cells lacking DNAJB6a adapt gain addiction to the oncogenic and tumor promotion supportive AKT signaling [36].

Another possible mechanism of DNAJB6's ability to counter metastatic spread might involve enhancement of cell adhesion through its interaction with urokinase-type plasminogen activator (uPA) receptor (uPAR). uPAR has been implicated in multiple cellular pathways, including proteolysis, cell adhesion and signal transduction. uPA and its receptor-dependent cell adhesion to the extracellular matrix protein, vitronectin, is an important event in cancer. The interaction between vitronectin and uPAR has also been implicated in regulating processes necessary for endothelial cell invasion and migration at vitronectin-rich extracellular matrix sites as well as in facilitating intracellular signaling. Functionally the interaction between uPAR and vitronectin can promote both, cellular adhesion and migration, and may direct uPAR to focal contacts. Bock *et al.* [10] identified that MRJ interacts functionally with uPAR to increase uPAR mediated cell adhesion to vitronectin, which was confirmed in breast cancer MDA-MB-231 cells. The exact mechanism of how MRJ regulates uPAR to increase adhesion to vitronectin remains to be defined. It has already been shown that the expression of uPAR in HEK293 cells leads to the formation of tight complexes with ß1 integrins to promote the adhesion of these cells to vitronectin. Role of the chaperone-co-chaperone duo was clearly evident in this regulation. Lin *et al* clearly demonstrated that HSP70 and DNAJB6 formed a triple complex with uPAR, indicating that uPAR is another client protein of DNAJB6 [78]. Mechanistic investigations revealed that DNAJB6 up-regulated phosphorylation of ERK1/2 and FAK suggesting that MAPK pathway was involved. These findings are critical towards providing added understanding of the roles of DNAJB6 in regulating cancer metastasis [78]. DNAJB6 was also found to directly interact with the intermediate filament keratin 18 (K18), and regulated K8/18 filament organization [79, 80]. Indeed, uPAR has also been found to interact with K18 [81], and DNAJB6 has the ability to direct K18 filaments to the proteasome. Thus these studies indicated a novel insight in offering a potential for the MRJ/uPAR interaction to modulate tumor growth by either altering keratin filament organization and/or promoting vitronectin binding *via* ß1 integrins. However, the specific roles of DNAJB6a *versus* b isoforms in this interaction remain to be elucidated.

Since DNAJB6 is down-regulated in cancers, knowledge about the factors responsible for its down-regulation are critical to understand the etiology of EMT and invasion in DNAJB6 deficient tumors. Investigations by Mitra *et al* demonstrated that miR-632 may function as a negative regulator for DNAJB6 expression. Invasive and metastatic breast cancer cells express high levels of miR-632 compared with mammary epithelial cells. In response to exogenous miR-632 expression, DNAJB6 protein levels are down-regulated and the resultant cell population shows significantly increased invasive ability. Silencing endogenous miR-632 abrogates invasive ability of breast cancer cells and promotes epithelial-like characteristics noted by E-cadherin expression with concomitant decrease in mesenchymal markers such as Zeb2 and Slug. It is noteworthy that there was an inverse trend noted for the expression of miR-632 and DNAJB6 [82]. However involvement of miR-632 in other cancers and pathologies in relation to DNAJB6 is still to be elucidated. It is also noteworthy that much remains to be described regarding the regulation of DNAJB6 gene and protein expression.

## THE FUNCTIONS OF SHORT ISOFORM OF DNAJB6 IN CANCER

As stated previously the long and short spliced variants of DNAJB6 have a significant identity. Thus it is logical to expect that the short form of DNAJB6 will also have a role in tumor biology. Unlike DNAJB6a which is predominantly located in the nucleus, DNAJB6b is predominantly located in the cytoplasm due to the lack of a C-terminal nuclear localization sequence (NLS). However, this short isoform is capable of translocating to the nucleus in response to heat shock and hypoxia [83]. The C-terminal sequence of DNAJB6b is critical for nuclear translocation; however this sequence does not show homology to any reported protein domains. Based on the identity of the amino acid sequences of DNAJB6 spliced variants, it can be expected that they may have significant redundancy in their functional capabilities. Cytoplasmic functions of MRJ(S) in relation to cancer biology are still to be defined. However, contrary to expectations, nuclear localization of DNAJB6b exhibits promotion of malignancy such as increased proliferation and invasiveness. The translocation of DNAJB6b to the nucleus and the ensuing tumor progression looks logical in the context of hypoxia, which is known to promote tumor growth, chemoresistance, invasiveness, and metastasis [84-87]. With tumor growth, the intratumoral microenvironment of a solid tumor becomes hypoxic and tumor cells show more aggressive properties [88]. The possible mechanism might be as follows; as the tumor grows, more and more cells become exposed to chronic levels of hypoxia, which may drive DNAJB6b to the nucleus and maintain it there, promoting proliferation, invasiveness and the further growth of the tumor. It will be very interesting to evaluate the levels of these two spliced variants with the tumor growth and evaluate their sub-cellular location and correlate that with prognosis of patients. It is conceivable that differential locations of these spliced isoforms of DNAJB6 and their loss may also contribute to the intra tumoral heterogeneity. Elaboration of such detailed aspects of DNAJB6 biology may be undertaken in future upon the development of antibodies specific to these isoforms.

## DNAJB6's FUNCTIONS IN EMBRYONIC DEVELOPMENT

It is an accepted notion that tumorigenesis and development shows erroneous manifestation of embryonic developmental signaling and events. Keeping this in mind, it is important to note the lessons revealed from the mouse model studies of DNAJB6.

DNAJB6 (murine: Mrj) has emerged as a key player in regulation of embryonic development. These important observations emerged from the study of MRJ knockout mouse. Mrj is widely expressed throughout the adult mouse however, during development of the embryo and it is essential for chorioallantoic attachment, a key developmental milestone required for mouse placenta development [32]. It mediates keratin turnover and prevents the formation of toxic inclusion bodies in trophoblast cells of the placenta. These inclusions in chorionic trophoblast cells cause cytotoxicity and disrupt chorion trophoblast cell organization that prevents chorioallantoic attachment [80]. It is also noted that Mrj(-/-) embryos exhibit neural tube defects independent of the placenta phenotype, including exencephaly and thin-walled neural tubes. The mechanistic details of these observations still remain to be described [33]. Further studies also revealed that cell-cell adhesion defects in Mrj mutant trophoblast cells are associated with failure to pattern the chorion during early placental development. Keratin aggregates found in Mrj(-/-) chorionic trophoblast cells are associated with abnormal cell morphology, collapse of the actin cytoskeleton, E-cadherin and β-catenin misexpression, and extracellular matrix (ECM) disorganization. Mrj(-/-) trophoblast cells *in vitro* are nonadherent and display erratic migratory behavior. This differentiation defect was not solely attributable to E-cadherin misexpression or ECM disorganization [89]. It seems logical to speculate that these observations in Mrj(-/-) embryos may be related to events in embryonic epithelial-mesenchymal-transition (Type I EMT) and bear similarity to the ones reported in cancer related EMT.

Related to studies in development and also possibly of relevance to its roles in cancer biology, DNAJB6 functions in cell division. As mentioned, DNAJB6 specifically interacts with Keratin18 (K18) suggesting that DNAJB6 may play an important role in the regulation of K8/18 filament organization as a K18-specific co-chaperone. Since the keratin and actin cytoskeletons are required to establish and maintain cell polarity, the collapse of the keratin cytoskeleton in Mrj(-/-) trophoblast cells may alter placement of the microtubule organizing center resulting in symmetric rather than asymmetric partitioning of cell fate factors [79, 89]. DNAJB6 has also been indicated in promoting cell cycle arrest. It is up-regulated in M-phase of HeLa cells. It is dispersed throughout the cell during late mitosis and localized in nucleolus during interphase, so the activity of DNAJB6 is regulated by its cell cycle specific expression together with its differential subcellular localization [90]. However, clear understanding of which form resides in which cellular compartment at what level in which stage of cell cycle in normal *vs* cancerous cells is still lacking. During cell division DNAJB6 stabilizes Schlafen1 (Slfn1). Slfn1 is a member of the Schlafen family playing an important role in the establishment and maintenance of quiescence in T-lymphocytes. Slfn1 moderates localization of DNAJB6 and enhances its cell-cycle-arrest-promoting function [7, 90]. However, clear definition of this activity in other cell types and disease situations has yet to emerge.

## CONCLUSIONS AND PERSPECTIVES

It is certainly evident that DNAJB6 has critical roles in development and organs or tissues of vital importance such as brain, heart and muscles (Figure 4). It regulates key cellular physiologic events such as cell division, cell polarity, cell morphology, stabilization or mediation of certain protein-protein interaction and down-regulation of unwanted protein inclusions. The lethal phenotype of the Mrj(-/-) mouse indicates a lack of redundancy of function in that other Hsp40 members do not substitute for DNAJB6 function. Thus it is not unexpected that DNAJB6 plays diverse roles in multiple pathologies.

Cancer is a disease which could partly be attributed to the failure of cellular checkpoints that ensure normal cellular homeostasis. Thus the involvement of DNAJB6 in suppression of tumorigenicity and metastasis is intuitive. However, investigations about the roles of DNAJB6 in tumor biology are still evolving. Relevance of signaling and molecular mechanisms influenced by DNAJB6 in other pathophysiologies and potential relevance of mutations in DNAJB6 also need to be investigated in malignant progression. Understanding the roles of spliced variants of DNAJB6 in tumor biology and the modulation of underlying signaling pathways is very critical. For example overtly in opposition to the observations of loss of (or reduced) expression in breast, melanoma and esophageal cancers, overexpression of DNAJB6 was found in 39% of the colorectal cancer (CRC) tissues. A positive correlation was observed from Kaplan-Meier survival analysis between DNAJB6 expression and overall survival [35]. Silencing of the DNAJB6 gene inhibited the invasion of CRC cells and was accompanied by a significant reduction in the protein levels of IQ-domain GTPase-activating protein 1 (IQGAP1) and phosphorylated ERK (pERK). *In vivo* assay showed that inhibition of DNAJB6 expression decreased the lung metastases of CRC cells. This data suggest that DNAJB6 plays an important oncogenic role in CRC cell invasion by up-regulating IQGAP1 and activating the ERK signaling pathway and that DNAJB6 may be used as a prognostic marker for CRC [35]. Though relevance of each spliced isoform of DNAJB6 still remains to be described CRC, it is conceivable that the signaling networks regulated through DNAJB6 are tissue specific and thus may remain cancer specific. Overall additional studies on DNAJB6 bear promising potential to unravel critical details in tumor progression and metastasis.

**Figure 4:** DNAJB6 is associated with various diseases and physiological processes

## Abbreviations and acronyms

APC: adenomatous polyposis coli
CBP: CREB-binding protein
CK1 α: casein kinase 1α
DKK1: dickkopf 1 homologue
Dvl: Dishevelled
DYRK1: dual-specificity tyrosine kinase 1
EMT: epithelial mesenchymal transition
EST: expressed sequence tag
GSK3β: glycogen synthase kinase 3β
HCMV: human cytomegalovirus
HDACs: histone deacetylases
HIV-2: human immunodeficiency virus type-2
HPD: Histidine-Proline-Aspartic acid
HSPA8: heat shock 70 kDa protein 8
Hsps: heat-shock proteins
K18: keratin 18
LRP5/6: low-density lipoprotein receptor-related protein5/6
MRJ: mammalian relative of DnaJ
MSX1: muscle segment homebox 1
NFAT: nuclear factor of activated T cells
NHR: N terminal homology region
NLS: nuclear localization sequence
OPN: osteopontin
PIC: preintegration complex
PKA: protein kinase A
PP2A: protein phosphatase 2, submit unit A
siRNA: small interfering RNA
Slfn1: schlafen1
TBP: TATA box binding protein
TCF/LEF: T-cell factor /lymphocyte enhancer factor
TNF-α: tumor necrosis factor α
uPA: urokinase-type plasminogen activator
uPAR: urokinase-type plasminogen activator receptor
